# Exploration of ACE-Inhibiting Peptides Encrypted in *Artemisia annua* Using *In Silico* Approach

**DOI:** 10.1155/2022/5367125

**Published:** 2022-05-23

**Authors:** Muhammad Naveed Shahid, Maryam Zawar, Adil Jamal, Bahaeldeen Babiker Mohamed, Sana Khalid, Fayez Saeed Bahwerth

**Affiliations:** ^1^Department of Botany, Division of Science and Technology, University of Education, Lahore, Pakistan; ^2^Sciences and Research, College of Nursing, Umm Al Qura University, Saudi Arabia; ^3^Institute of Environment Natural Resources, The National Centre of Research, Khartoum, Sudan; ^4^Department of Botany, Lahore College for Women University, Lahore, Pakistan; ^5^Central Laboratory and Blood Bank, King Faisal Hospital, Makkah-24235, Saudi Arabia

## Abstract

The renin-angiotensin system (RAS) is involved in body fluid regulation, but one of its enzymes, angiotensin-converting enzyme (ACE), indirectly causes hypertension by constricting blood vessels. Autoimmune illness is linked to the increased risk of hypertension and cardiovascular disease. In this study, ACE-inhibiting peptides were studied from *Artemisia annua* proteins. *In silico* hydrolysis of proteins was performed by BIOPEP-UWM using proteolytic enzymes from plant, microbial, and digestive sources. The physicochemical properties of 1160 peptides were determined using the peptide package of R studio. Di- and tripeptides were mostly released with a molecular weight of 170 to 350 Da. PeptideRanker was used to select 16 peptides from a pool of 1160 peptides based on their likelihood of being bioactive. Molecular docking was performed by DS 2020 and AutoDock Vina, which revealed that the stability of the ligand-receptor complex is due to hydrogen bonding and electrostatic and hydrophobic interactions. Their binding energies ranged from -31.81 to -20.09 kJ/mol. For drug-likeness evaluation, an online tool SwissADME was used that follows the ADME rule (absorption, distribution, metabolism, and excretion) to check the pharmacokinetics and drug-likeness of the compound. In the future, the released peptides can be used to make functional nutraceutical foods against hypertension.

## 1. Introduction

Most cardiovascular diseases caused by hypertension have a high death ratio, and approximately 66% of hypertension cases are found, especially in developing countries [1]. Autoimmune illnesses, such as systemic lupus erythematosus and rheumatoid arthritis, are linked to an increased risk of hypertension and cardiovascular disease [2]. A major community-based research, for example, discovered a higher prevalence of hypertension among RA patients (31%), compared to the general population (23%) [3]. A hormone system renin-angiotensin system (RAS) is involved in body fluid regulation but indirectly increases blood pressure [4]. Angiotensin-converting enzymes in the RAS system convert angiotensin *Ι* to angiotensin *ΙΙ*, which narrows the blood vessels and causes hypertension [5]. From different natural resources, many ACE-inhibiting peptides have been studied to stabilize blood pressure [6].

As the frequency of hypertension increased day by day, antihypertensive activity of most of the bioactive peptides was studied and gained much attention [7]. For the inhibition of ACE, many antihypertensive drugs have been discovered, such as captopril, lisinopril, and aliskiren. On the one hand, these drugs are beneficial, but at the same time, they cause serious side effects, such as disturbing the potassium level, loss of taste, and dizziness [8]. Therefore, antihypertensive peptides were studied from different sources, such as chia seeds, sesame seeds, and flaxseeds.

By hydrolysis of mung bean proteins, five ACE-inhibiting peptides (LPRL, YADLVE, LRLESF, HLNVVHEN, and PGSGCAGTDL) were released, and their effect was studied when given to hypertensive rats. The results showed that YADLVE was more effective than others [9]. Banana pulp was purified into three protein extracts as purified, partially purified, and crude. Upon hydrolysis with proteolytic enzymes, the crude extract released more ACE-inhibiting peptides (85.20%) [10].

Liang et al. [11] identified a peptide IAF from pumpkin seeds using *in silico* approaches. By molecular docking, a strong interaction was found between IAF and ACE, which shows hydrogen bonding between two residues of ACE, His513 and Glu162, with IAF. Similarly, many antihypertensive peptides are released from different plant sources, such as bitter melon seeds [12], peach seeds [13], cottonseed [14], hemp seeds [15], sesame seeds [16], and date seeds [17].

Four novel ACE-inhibiting peptides (MAF, NMF, HPF, and MCG) were identified from quinoa proteins. Hydrolysis of proteins was performed by an *in silico* method using plant proteolytic enzymes, ficin, papain, and stem bromelain [18]. *Artemisia annua* is a short-day plant containing a high protein content and several essential amino acids. Due to high antimalarial activity, the Nobel Prize was awarded to the species in 2015 [19].

In this research, antihypertensive peptides were studied from *A. annua* proteins using bioinformatics tools. A molecular docking study revealed the stability of the peptide and ACE complex. These peptides act as inhibitors of angiotensin-converting enzyme (ACE). The released peptides are then incorporated into food products to make functional foods.

## 2. Materials and Methods

### 2.1. Hydrolysis of Proteins by Proteolytic Enzymes

Proteins were selected on the basis of secondary metabolite synthesis, and for sequence retrieval, the UniProt database (https://www.uniprot.org/) was used. The BIOPEP-UWM database [20] (http://www.uwm.edu.pl/Biochemia/Index.Php/En/Biopep) was used to hydrolyze the proteins by different proteolytic enzymes. Nine types of proteases from three sources were used: plant proteases (papain, ficin, and stem bromelain), digestive enzymes (pancreatic elastase *ΙΙ*, pepsin, and trypsin), and microbial enzymes (subtilisin, thermolysin, and proteinase P1). After hydrolysis, ACE-inhibiting peptides were selected using the BIOPEP-UWM “search for active fragment” feature.

### 2.2. Physiochemical Parameters of ACE Inhibitory Peptides Released by Proteolytic Enzymes

Using the “peptides” package in RStudio [21], the physicochemical properties of the released peptides were studied. The properties include molecular weight, net charge, isoelectric point, hydrophobicity, and Boman index.

### 2.3. Molecular Docking of Antihypertensive Peptides with ACE Receptor

From released ACE inhibitory peptides, only 16 peptides were selected for molecular docking using the PeptideRanker tool (http://distilldeep.ucd.ie/PeptideRanker/). These 16 peptides with the inhibitory drug captopril were used as ligands, and their structures were generated using Discovery Studio 2020 (https://discover.3ds.com/discovery-studio-visualizer-download). Human ACE structure was used as receptor for docking. AutoDock Vina [22] was used to prepare the receptor by removing the water molecules and adding charges to the protein. For ligand binding, a site was constructed (radius 13 Å; coordinates *x*: 38.7154, *y*: 35.4135, and *z*: 41.6065).

For docking result visualization, Discovery Studio 2020 was used, and hydrogen bonding and electrostatic and hydrophobic interactions were studied between the ligand and receptor residues.

### 2.4. Evaluation of Drug-Like Properties of Peptides

The drug-like properties of peptides were evaluated *in silico* using SwissADME (http://www.swissadme.ch). This tool follows the ADME rule (absorption, distribution, metabolism, and excretion) to check the pharmacokinetics and drug-likeness of compounds. ToxinPred (http://crdd.osdd.net/raghava/toxinpred/) was used to predict the toxicity of compounds.

## 3. Results

### 3.1. Proteolytic Enzyme Sources and Effect on Antihypertensive Peptides

A total of 11 proteins of *Artemisia annua* were selected, and their characteristics are shown in Table 1. On hydrolysis, most of the released peptides were di- and tripeptides. The number of released peptides depends on the enzyme source and type (Table 2). A total of 1160 ACE inhibitory peptides were released, from which 631, 141, and 388 were released by plant, digestive, and microbial proteases, respectively. Approximately 54.3% of peptides were released by plants, of which 32.3%, 28%, and 40% were released by enzymes, papain, stem bromelain, and ficin, respectively. Microbial proteases release 33.4% of ACE inhibitory peptides with a high degree of hydrolysis by thermolysin (36.3%), proteinase P1 (21.3%), and subtilisin (42.2%). However, fewer peptides were released by digestive enzymes (12.2%) than by the other two types. For trypsin, pepsin, and pancreatic elastase *ΙΙ*, the degree of hydrolysis was 14.8%, 36%, and 49%, respectively. The number of peptides revealed that plant proteases were superior to microbial and digestive enzymes.

### 3.2. Physiochemical Parameters of ACE Inhibitory Peptides Released by Proteolytic Enzymes

The physiochemical parameters of ACE-inhibiting peptides that have been released by hydrolysis were demonstrated (Figure 1). The molecular weight varies between 170 and 410 Da. The molecular weights of dipeptides ranged from 170 to 350 Da, and they were abundantly released from proteins. The MW of the majority of the dipeptides ranged between 250 and 300 Da. Tripeptides ranging in size from 300 to 410 Da were also found (Figure 1(a)). The isoelectric point of peptides ranged from 3.8 to 12.5, and approximately 212 peptides had a pI less than 5 with a net charge of -1, which indicates the presence of amino acids with negative charges in most of the peptides.

Approximately 790 peptides had pI ≤ 8 with a net charge of zero, while 180 peptides had pI ≤ 11 with a net charge of 1. These peptides mostly contain amino acids with positive charges (Figures 1(b) and 1(c)). The hydrophobicity of the 1160 peptides ranged from -3.50 to 5.00. Approximately 494, 196, and 410 peptides were neutral, hydrophilic, and hydrophobic, respectively (Figure 1(d)). The ACE inhibitory peptide Boman index ranged from -3.62 to 14.92, and most of the peptides had BI less than 2 (Figure 1(e)).

### 3.3. Molecular Docking of Antihypertensive Peptides with ACE Receptor

The probability of peptides' bioactivity was predicted by PeptideRanker using score values ranging from 0.021 to 0.99. The first 16 peptides with a probability value close to 1 were selected for docking. The binding energies of the ligand-receptor complex ranged from -31.81 to -20.09 (Table 3). According to the results, most of the peptides showed strong hydrogen bonding as well as electrostatic and hydrophobic interactions with ACE residues (Asn70, Val518, His513, Thr140, and Phe512), which showed the ACE-inhibiting properties of peptides (Figure 2). RF and RW interacted with ACE active site pockets as S1 and S2, respectively.

GW interacted with Asp141, Val148, and Ile73 via hydrogen bonding and hydrophobic interactions. Hydrophobic amino acids of peptides, present near the C-terminus, strongly interact with active site residues. Hydrogen bonds were displayed (Table 4) that are found in ligand-receptor complexes. His348, Glu372, and His344 coordinates interact with the zinc ion present in the ACE structure, showing the importance of Zn in ACE inhibition. As none of the peptides interacted with Zn ions, peptides showed low inhibitory activity compared to captopril (Table 3).

### 3.4. Drug-Likeness Evaluation

The peptide drug-likeness profile was demonstrated (Table 5). The results revealed numerous similarities of peptides when compared to the inhibitory drug captopril. As the number of ROTB and TPSA of RF, RW, and FP peptides were not according to the required value, they were present outside the estimated range (see the shaded region in Figure 3).

All of the other peptides had the same bioavailability as captopril (0.55). None of the peptides showed CYP3A4 inhibition except for RF, RW, and FR, and all the peptides also had a high GIA. Except for MW and WL, all other peptides acted as P-glycoprotein substrates and had high bioavailability and GIA.

## 4. Discussion

For the breakdown of peptide links in proteins, proteolytic enzymes (also known as proteases or proteinases) were used. Because of their critical roles in biological processes, they are vital in medicine, pharmaceuticals, biotechnology, and a variety of research applications, such as protein digestion, peptide synthesis, cell culture, and peptide sequencing [23]. The amino acid specificity at both terminals determines the type of protease used for peptide synthesis [24]. As most ACE inhibitory peptides consist of 2-12 amino acids, the binding of peptides with ACE residues becomes very easy [25].

This is due to the wide range of specificity of amino acids, such as papain, which primarily cleaves hydrophobic and basic amino acids [23]. The peptide's affinity for ACE was increased when positively charged amino acids and basic amino acids were present at the C and N termini, respectively. As a result, antihypertensive activity also increased [26].

The hydrophobicity of amino acid side chains typically depends on the molecular weight of the peptides [27]. Amino acid hydrophobicity at the C-terminus influences ACE inhibition activity, as higher hydrophobicity directly increases the inhibition action [28]. Most of the dipeptides had high hydrophobicity at the C-terminus; therefore, the inhibition action of peptides increased [29]. Hydrogen bonding plays an important role in the structure of ligand-receptor complexes [30].

Coordination with other residues, on the other hand, caused distortion of Zn ions, due to which ACE lost its inhibitory action [31]. The optimized cutoff values for molecules being permeable have been proposed, which include PSA < 140, ClogP < 5, HBA < 10, HBD < 5, and MW < 350 [32]. By following these optimized values, the oral administration properties of molecules increased [33]. The flexibility and polarity of the drugs affect their oral bioavailability. The number of ROTB and TPSA represents the flexibility and polarity of a compound. The oral bioavailability of a compound becomes low and high due to the presence of more rotatable bonds and small topological surface areas, respectively [34].

ACE inhibitors are partially metabolized by CYP3A4 because they have little effect on cytochrome interactions [35, 36]. The CYP3A5 enzyme family is important in drug metabolism [37]. Interactions between drug-active compounds and any of the CYP isozymes can result in drug bioaccumulation (when a CYP isozyme is activated) or rapid metabolism (when a CYP isozyme is inhibited) in the body. Both scenarios are undesirable because the first can result in overdosing and the second in toxicity [38].

ACE inhibitors are routinely given for the treatment of hypertension and renal dysfunction in systemic lupus erythematosus (SLE) patients, despite the fact that no randomised controlled studies have been conducted [39]. The use of ACE inhibitors during SLE is generally well tolerated and associated with a delay in the onset of renal involvement and a decrease in the risk of disease relapse in SLE patients, which is likely due to a decrease in angiotensin II as well as the immunomodulatory effect of renin-angiotensin system blockade [40]. As a result, in individuals with autoimmune illness, RAS blockage may have a dual impact in controlling the autoimmune disease and its accompanying hypertension [41].

## 5. Conclusion

*Artemisia annua* proteolytic enzymes (papain, ficin, and stem bromelain) produced more antihypertensive peptides than microbial (thermolysin, proteinase P1, and subtilisin) and digestive (trypsin, pepsin, and pancreatic elastase I) enzymes. In molecular docking, a stable interaction between ligands and receptors by hydrogen bonding was studied. In addition, *in silico* drug-likeness evaluation of the ACE-inhibiting peptides revealed that all peptides followed at least four of the five rules of Lipinski filters, but FR, RW, and RF violated one of the rules. As peptides are released from proteins of medicinal plants through proteolytic enzyme hydrolysis, therefore they are used in therapeutic settings and have the ability to improve food products by being used as nutraceuticals.

## Figures and Tables

**Figure 1:** Physiochemical parameters of ACE-inhibiting peptides: (a) molecular weight, (b) isoelectric point, (c) net charge, (d) hydrophobicity, and (e) Boman index.

**Figure 2:** The best pose of ligand docked with receptor showing hydrogen bonding as well as hydrophobic and electrostatic interaction.

**Figure 3:** Oral bioavailability range of the ACE-inhibiting peptides and inhibitory drug (captopril). LIPO: lipophilicity (ClogP_o/w_ < 5); SIZE: molecular size (mol < 500 g/mol); INSOLU: solubility; POLAR: polarity (TPSA < 130 Å^2^); log S (ESOL) < 6; INSATU: insaturation (fraction Csp3 < 1); FLEX: flexibility (number of rotatable bonds < 9). The colorful zone represents the optimum physicochemical space for oral bioavailability.

**Table 1:** List of selected proteins and their attributes.

S. no.	Accession no.	Protein	Function	Residue length	MW (kDa)
1	Q9LLR9	Epi-cedrol synthase	Terpenoid biosynthesis	547	63.57
2	Q9SPN0	R-linalool synthase QH1, chloroplastic	Terpenoid biosynthesis	567	65.71
3	Q8SA63	Beta-caryophyllene synthase	Sesquiterpene biosynthesis	548	63.75
4	Q94G53	(-)-*beta*-Pinene synthase, chloroplastic	Monoterpene biosynthesis	582	67.52
5	Q1PS23	Amorpha-4,11-diene 12-monooxygenase	Antimalarial endoperoxide artemisinin biosynthesis	495	55.72
6	Q9AR04	Amorpha-4,11-diene synthase	Antimalarial endoperoxide artemisinin biosynthesis	546	63.94
7	Q43319	3-Hydroxy-3-methylglutaryl coenzyme A reductase	Isoprenoid biosynthesis	560	60.34
8	Q9SWQ3	Hydroxymethylglutaryl-CoA reductase (NADPH)	Isoprene biosynthesis	567	61.7
9	C5H429	Artemisinic aldehyde delta(11(13)) reductase	Antimalarial endoperoxide artemisinin biosynthesis	388	42.59
10	C5I9X1	Aldehyde dehydrogenase 1	Sesquiterpene biosynthesis	499	53.8
11	P49350	Farnesyl pyrophosphate synthase	Sesquiterpene biosynthesis	343	39.41

**Table 2:** The source of the enzyme, type of enzyme, and released ACE inhibitory peptides by each enzyme are listed.

Enzyme source	Enzyme type	Total no. of ACE-inhibiting peptides
Plant	Papain	204
	Ficin	252
	Stem bromelain	175
Microbial	Thermolysin	141
	Subtilisin	164
	Proteinase P1	83
Digestive	Trypsin	21
	Pepsin	51
	Pancreatic elastase *ΙΙ*	69
Total		1160

**Table 3:** Evaluated binding energies and Zn *ΙΙ* coordination distances of ligand-receptor complexes.

Ligand	Affinity energy (kJ/mol)	Zn coordination	
		Distance (Å)	Atom
AF	-26.98		No zinc coordination
FG	-26.79		No zinc coordination
FP	-23.02		No zinc coordination
FY	-31.81		No zinc coordination
FR	-25.12		No zinc coordination
GW	-22.19		No zinc coordination
LW	-28.47		No zinc coordination
MW	-23.02		No zinc coordination
RF	-30.98		No zinc coordination
RW	-27.44		No zinc coordination
WG	-28.88		No zinc coordination
WL	-24.28		No zinc coordination
YF	-28.28		No zinc coordination
CF	-27.95		No zinc coordination
GF	-20.09		No zinc coordination
MF	-21.35		No zinc coordination
Captopril	-26.78	2.76	Sulfhydryl group of captopril

**Table 4:** In the best docking pose of the ligand-receptor complex, hydrogen bonds and their distances (Å) with ACE residues are shown.

ACE residues in H-bonding	Number of H-bonds and their corresponding distance (Å)																Captopril
	FG	FP	AF	FR	FY	GW	LW	RF	RW	WG	MW	WL	YF	CF	GF	MF	
THR144:OG1		1 (2.7)		1 (2.1)					1 (2.6)			1 (3.7)	1 (1.9)		1 (2.0)	1 (2.0)	
TYR2:O					2 (2.1, 2.3)												
ASN70:OD1	1 (3.3)		1 (1.9)				1 (2.6)			1 (1.9)							1 (2.8)
LEU140:O				1 (3.0)				2 (2.9, 2.5)					1 (2.7)		1 (2.6)	1 (3.0)	1 (3.7)
ILE73:O				1 (2.6)		1 (2.3)						1 (2.5)					
SER516:O	2 (2.7, 2.9)				1 (2.3)					1 (2.2)				1 (2.0)			1 (3.3)
PHE1:O	1 (2.1)	1 (3.0)		1 (3.6)				1 (2.2)							1 (3.3)	1 (2.9)	
TRP2:O						1 (3.8)					2 (3.4)						
ARG1:O									1 (2.8)								
PRO515:O		1 (2.4)															
GLU143:OE1	1 (2.5)		1 (2.1)		1 (2.7)												1 (3.6)
LEU1:O							1 (2.4)					1 (3.6)					
THR75:O				1 (2.6)					2 (2.4, 2.0)					1 (2.0)			
TYR523:OH		1 (2.0)						1 (2.6)						1 (2.6)			
ASN66:OD1			1 (3.2)				1 (2.5)			1 (3.0)							1 (2.2)
SER78:OG												2 (2.3, 2.4)	1 (2.5)		1 (2.5)	2 (3.6, 2.8)	
TRP2:OXT				1 (3.8)		1 (3.0)	1 (3.0)		1 (2.3)		1 (3.8)						
HIS513:NE2	1 (2.4)		2 (2.5, 3.0)					1 (2.1)									
ASP141:OD1												1 (2.5)		1 (2.3)			
Total	6	4	5	6	4	3	4	5	5	3	3	6	3	4	4	5	5

**Table 5:** *In silico* drug-likeness assessment illustrating the antihypertensive peptide ADMET profile.

	Physicochemical properties					Toxicity	Lipophilicity		Drug-likeness		Pharmacokinetics		
	Mol. wt. (g/mol)	ROTB (*n*)	HBA (*n*)	HBD (*n*)	ESOL log S	ToxinPred (SVM score)	TPSA (Å)	ClogP_o/w_	Bioavailability score	Lipinski filer	GIA	P-glycoprotein substrate	CYP3A4 inhibitor
Rule	<500	<10	<10	<5	—	—	<140	<5	—	—	—	—	—
AF	236.27	6	4	3	0.39 (HS)	Nontoxic -0.8	92.42	0.05	0.55	Yes (0)	High	No	No
FG	222.24	6	4	3	0.48 (HS)	Nontoxic -0.8	92.42	-0.16	0.55	Yes (0)	High	No	No
FP	262.3	5	4	3	-0.51 (VS)	Nontoxic -0.8	83.63	0.32	0.55	Yes (0)	High	No	No
FR	321.37	11	5	6	0.79 (HS)	Nontoxic -0.8	154.32	-0.66	0.55	Yes (1)	Low	No	No
FY	328.36	8	5	4	-0.66 (VS)	Nontoxic -0.8	112.65	0.83	0.55	Yes (0)	High	No	No
GW	261.28	6	4	4	0.23 (HS)	Nontoxic -0.8	108.21	-0.18	0.55	Yes (0)	High	No	No
LW	317.38	8	4	4	-0.18 (VS)	Nontoxic -0.79	108.21	1.09	0.55	Yes (0)	High	No	No
MW	335.42	9	4	4	-0.67 (VS)	Nontoxic -0.8	133.51	0.86	0.55	Yes (0)	High	Yes	No
RF	321.37	11	5	6	0.77 (HS)	Nontoxic -0.8	154.32	-0.59	0.55	Yes (1)	Low	No	No
RW	360.41	11	5	7	0.26 (HS)	Nontoxic -0.8	170.11	-0.44	0.55	Yes (1)	Low	No	No
WG	261.28	6	4	4	-0.11 (VS)	Nontoxic -0.8	108.21	0.08	0.55	Yes (0)	High	No	No
WL	317.38	8	4	4	-1.11 (VS)	Nontoxic -0.8	108.21	1.13	0.55	Yes (0)	High	Yes	No
YF	328.36	8	5	4	-0.66 (VS)	Nontoxic -0.8	112.65	0.78	0.55	Yes (0)	High	No	No
CF	268.33	7	4	3	0.32 (HS)	Nontoxic -0.79	131.22	-0.02	0.55	Yes (0)	High	No	No
GF	222.24	6	4	3	0.32 (HS)	Nontoxic -0.8	92.42	-0.23	0.55	Yes (0)	High	No	No
MF	296.39	9	4	3	-0.25 (VS)	Nontoxic -0.8	117.72	0.72	0.55	Yes (0)	High	No	No
Captopril	217.29	4	3	1	-1.14 (VS)		96.41	0.62	0.56	Yes (0)	High	No	No

## Data Availability

All data is available in the main manuscript.
